The article "Serum ICAM-1 as a Predictor of Prognosis in Patients with Acute Ischemic Stroke" was published in 2021. Journal: Biomed Res Int.

# Serum ICAM-1 as a Predictor of Prognosis in Patients with Acute Ischemic Stroke

**DOI:** 10.1155/2021/5539304

**Published:** 2021-03-18

**Authors:** Lei Wang, Yan Chen, Depeng Feng, Xiaoling Wang

**Affiliations:** ^1^Department of Infectious Disease, Beijing Tiantan Hospital, Capital Medical University, Beijing, China; ^2^Department of Geriatric Medicine, Shandong Provincial Third Hospital, Cheeloo College of Medicine, Shandong University, Jinan, Shandong Province, China; ^3^Department of Neurology, Liaocheng People's Hospital, Liaocheng, Shandong Province, China

## Abstract

**Objective:**

Inflammation is one of the key mechanisms involved in functional impairment after stroke. Intercellular adhesion molecule-1 (ICAM-1) is an important inflammatory molecule in the body. The purpose of our study was to determine the correlation between ICAM-1 and the prognosis of acute ischemic stroke (AIS).

**Methods:**

286 AIS patients treated at Beijing Tiantan Hospital were continuously included in the study. The demographic data of the patients were collected, and the fasting blood within 24 hours of admission was collected to detect the clinical indicators. The functional prognosis was measured using the modified Rankin Scale (mRS) 3 months after stroke. The poor prognosis is defined as mRS ≥ 3. The enzyme-linked immunosorbent assay (ELISA) was used to determine the serum ICAM-1 levels.

**Results:**

The serum ICAM-1 levels of patients with poor prognosis were significantly higher than that of patients with good prognosis (144.2 ± 14.8 vs 117.5 ± 12.1 pg/ml). Receiver operating characteristic curve (ROC) analysis showed that the sensitivity and specificity of serum ICAM-1 for predicting the prognosis of AIS were 74% and 76%, respectively. In logistic regression analysis, the serum ICAM-1 level is still an independent predictor of poor prognosis (odds ratio [OR]: 0.52; 95% confidence interval [CI]: 0.318-0.839).

**Conclusions:**

Higher serum ICAM-1 levels on admission in AIS patients might increase the risk of poor prognosis.

## 1. Introduction

The definition of stroke is a neurological impairment syndrome caused by the permanent brain, spinal cord, or retinal cell death caused by vascular etiology [1]. The morbidity and disability rate of stroke are relatively high, with 13.7 million new stroke patients every year, and 5.8 million deaths due to stroke [2]. In the world, more than 80 million people have survived strokes, of which about 70% are ischemic strokes, and the rest are cerebral hemorrhage (ICH) or subarachnoid hemorrhage (SAH). Stroke is the second leading cause of death in the world, while it ranks first in China. China's national research and regular government reports show that the burden of stroke is high and is gradually increasing [3]. The pathogenic mechanism of AIS is complicated, and there is no cure [4, 5]. Therefore, finding the pathogenic target of AIS and developing targeted treatment are urgent problems to be solved.

The article "Serum ICAM-1 as a Predictor of Prognosis in Patients with Acute Ischemic Stroke" was published in 2021. Journal: Biomed Res Int.

Intercellular adhesion molecule-1 (ICAM-1), also named CD54, is a type I transmembrane protein with a molecular weight between 80 and 114 kDa, and its molecular weight varies depending on the level of glycosylation [6]. The full length of ICAM-1 consists of five immunoglobulin (Ig) domains, a short cytoplasmic tail with multiple threonine residues, and a transmembrane domain [7]. Alternative splicing is a common post transcriptional mechanism that is widely used to regulate the gene expression [8]. ICAM-1 can produce soluble ICAM-1 through alternative splicing, which can be measured in various body fluids [9]. Studies have shown that ICAM-1 levels are elevated in atherosclerosis, cardiovascular disease, and metabolic vascular neuropathy [10–13]. However, there are still few studies on the correlation between ICAM-1 and AIS.

Neurons, microglia, astrocytes, and vascular components together form a functional neurovascular unit, which is the anatomical basis for the pathogenesis of AIS [14, 15]. Microglia are important innate immune cells in the body, and their different activation states exert different inflammatory effects [16–18]. More and more evidences show that inflammation plays a key role in the pathogenesis of AIS and may become a potential target for treatment [19, 20]. In this study, we explored the predictive effect of the inflammatory molecule ICAM-1 on the prognosis of AIS, which may provide an important target for the therapeutic intervention of stroke.

## 2. Methods

### 2.1. Study Population

From January 2020 to December 2020, AIS patients who were treated at Beijing Tiantan Hospital were included in the study. After screening, a total of 286 patients were included in the study. An AIS attack is defined as the patient's first neurological deficit, which is confirmed by brain CT or MRI. The exclusion criteria include (1) past history of stroke, (2) combined with tumor, (3) combined with infectious disease or autoimmune disease, (4) intravenous thrombolysis or arterial thrombectomy, and (5) combined with cerebral hemorrhage. The study complied with the Declaration of Helsinki and was approved by the local medical ethics committee. Research subjects or guardians agree to participate in the research and sign an informed consent form.

### 2.2. Characteristics of AIS Patients

All subjects underwent the National Institute of Health Stroke Scale immediately after enrollment to evaluate the patients' neurological function. Their demographic data (age and gender) were collected. At the same time, the past medical history (hypertension, diabetes, coronary heart disease, and atrial fibrillation) was asked and recorded. An electronic sphygmomanometer is used to measure the patient's blood pressure in a quiet state. The patient's fasting blood glucose and total cholesterol were measured in the biochemical laboratory.

The article "Serum ICAM-1 as a Predictor of Prognosis in Patients with Acute Ischemic Stroke" was published in 2021. Journal: Biomed Res Int.

### 2.3. Serum ICAM-1 Determination

Fasting blood of all patients was collected within 24 hours of admission. Peripheral blood was allowed to stand for half an hour at room temperature and then centrifuged at low temperature and high speed. Separate and pack the serum and store it in a refrigerator at -80°C for later use. The concentration of serum ICAM-1 was determined by the enzyme-linked immunosorbent assay (ELISA). All ICAM-1 antibodies for the experiment were purchased from Abcam Co., Ltd. (Abcam, Cambridge, MA). The ELISA test method refers to the previous literature and product instructions [21–23].

### 2.4. Prognosis Assessment and Grouping

The modified Rankin Scale (mRS) is a commonly used neuroevaluation scale, mainly used to evaluate the degree of disability in patients with neurological dysfunction. The scale was first proposed by Dr. John Rankin of Scotland in 1957, and it has become the most widely used clinical outcome tool in stroke clinical trials [24–26]. In this study, the modified Rankin Score (mRS) was used to measure the functional prognosis 3 months after stroke. A good prognosis is defined as mRS < 3, and a poor prognosis is defined as mRS ≥ 3. According to the difference of mRS scores, AIS patients were divided into the good outcome group and poor outcome group.

### 2.5. Statistical Analysis

Continuous variables were described as mean ± standard deviation or median and interquartile range and compared with Student's *t*-test. Categorical variables are described as *n* (%) and compared with the chi-square test. The receiver operating characteristic curve is applied to determine the cut point of ICAM-1 to distinguish between good and poor outcomes. Logistic regression analysis was used to evaluate the independent contribution of different variables to prognosis prediction. Statistical analysis was performed using SPSS22.0 software (SPSS Inc., Chicago, Illinois, USA), and *p* value <0.05 was considered statistically significant.

## 3. Results

### 3.1. Characteristics of AIS Patients

A total of 286 AIS patients were included in this study. According to the mRS score, they were divided into a good outcome group (*n* = 181) and a poor outcome group (*n* = 105). The ages of AIS patients in the good outcome group and poor outcome group were (61.4 ± 8.9) and (61.7 ± 9.6) years, respectively. The proportion of men with AIS in the good outcome group and poor outcome group was 60.8% and 59.0%, respectively. There was no significant statistical difference in age and gender between the two groups (*p* > 0.05). We further compared the past medical history of the two groups of AIS patients, and we found that their incidence of hypertension, diabetes, coronary heart disease, and atrial fibrillation was not significantly different (*p* > 0.05). Regarding clinical indicators, such as systolic blood pressure, diastolic blood pressure, fasting blood glucose, and total cholesterol, there was also no significant statistical difference between the two groups (*p* > 0.05). However, the serum ICAM-1 concentrations of AIS patients in the good outcome group and the poor outcome group were (117.5 ± 12.1) and (144.2 ± 14.8) pg/ml, respectively, and the serum ICAM-2 levels of AIS patients in the poor outcome group were significantly higher in the good outcome group (*p* < 0.001). The characteristics of all AIS patients are shown in Table 1.

The article "Serum ICAM-1 as a Predictor of Prognosis in Patients with Acute Ischemic Stroke" was published in 2021. Journal: Biomed Res Int.

### 3.2. ROC Analysis for the Serum ICAM-1 Level in the AIS Patients

As shown in Figure 1, in order to evaluate the diagnostic value of serum ICAM-1 as a potential prognostic marker of AIS, we performed ROC curve analysis. For serum ICAM-1, the sensitivity is 74%, the specificity is 76%, and the area under the curve (AUC) is 0.772. The best cutoff value of the ROC curve for distinguishing good outcomes from poor outcomes is 129.5 pg/ml. When the baseline serum ICAM-1 concentration is higher than 129.5 pg/ml, it indicates that the prognosis of AIS patients is poor. However, when the baseline serum ICAM-1 concentration is lower than 129.5 pg/ml, it indicates that AIS patients have a good prognosis.

### 3.3. Logistic Regression Analysis

The clinical baseline characteristics were incorporated into logistic regression to analyze the predictive value of different variables on the prognosis of AIS. Clinical baseline characteristics include age, gender, NHISS score, hypertension, coronary heart disease, diabetes, atrial fibrillation, systolic blood pressure, diastolic blood pressure, fasting blood glucose, total cholesterol, and serum ICAM-1 concentration. The results of the logistic regression analysis are shown in Table 2. The results showed that after adjusting for age, gender, NHISS score, hypertension, coronary heart disease, diabetes, atrial fibrillation, systolic blood pressure, diastolic blood pressure, fasting blood glucose, and total cholesterol, the serum ICAM-1 level is still the prognosis of AIS patients' independent predictor (*p* = 0.007).

The article "Serum ICAM-1 as a Predictor of Prognosis in Patients with Acute Ischemic Stroke" was published in 2021. Journal: Biomed Res Int.

## 4. Discussion

The main finding of our current study is that the serum ICAM-1 levels of patients with poor AIS outcomes are significantly higher than those with good outcomes. Our further ROC analysis indicated that the cut-off value of serum ICAM-1 as a diagnostic target for predicting the prognosis of AIS was 129.5 pg/ml, and its sensitivity and specificity were 74% and 76%, respectively. After adjusting the clinical baseline data, the serum ICAM-1 level can still be used as an independent biomarker for predicting the prognosis of AIS patients.

Inflammation is the main factor affecting the pathobiology and prognosis of AIS [27]. Although the inflammatory response begins with local occlusion and hypoperfusion of blood vessels and ischemic brain parenchyma, the inflammatory mediators generated in situ spread throughout the organism, leading to systemic inflammation [28]. Increased blood levels of systemic inflammatory markers are associated with adverse outcomes after AIS. Animal studies have demonstrated the causal relationship between systemic inflammation and AIS neurological damage and poor prognosis [29]. The underlying mechanisms of systemic inflammation affecting the poor prognosis of AIS include neutrophil infiltration, blood-brain barrier (BBB) destruction, and cerebral ischemia-reperfusion injury [30, 31]. Animal experiments showed that reducing leukocyte infiltration could reduce the neurological damage of AIS and delay disease progression [32]. However, clinical trials of antileukocyte therapy have not reached a consistent conclusion with animal experiments.

ICAM-1 is a glycoprotein adhesion receptor mainly expressed on the surface of endothelial cells [33, 34]. Its main function is similar to chemokines and can induce the recruitment of leukocytes from the circulation to the inflammation site [35]. The unique domain of ICAM-1 allows it to be used as a biosensor, which can associate with the actin cytoskeleton after binding to a ligand to achieve signal transduction [36]. sICAM-1 is produced as a splice isoform of ICAM-1 or as a result of proteolytic cleavage. sICAM-1 retains all 5 extracellular Ig domains, and the molecular composition of the Ig domain of sICAM-1 varies depending on the protease that catalyzes the cleavage [9]. Studies have found that sICAM-1 has the dual effects of proinflammatory and anti-inflammatory [37], which suggests the complexity of its involvement in pathogenic mechanisms.

The mechanism of ICAM-1 involved in neuroinflammatory injury after stroke has been reported. Research by Zhang et al. showed that anti-ICAM-1 antibody could significantly reduce ischemic brain damage after focal cerebral ischemia in rats, while reducing polymorphonuclear leukocytes in the injured area [38]. Consistent with the above results, Bowes et al. further verified that anti-ICAM-1 could reduce neurological damage after stroke in a rabbit cerebral ischemia model, but it had no synergistic effect with tissue plasminogen activator (tPA) [39]. However, there are also different conclusions in animal experiments. Studies have shown that ICAM-1 knockout mice can neither inhibit the recruitment of neutrophils after cerebral ischemia nor can they provide protection for neurons after ischemia and reperfusion [40]. These different conclusions precisely suggest that ICAM-1 is involved in the complexity of inflammatory damage after stroke.

The article "Serum ICAM-1 as a Predictor of Prognosis in Patients with Acute Ischemic Stroke" was published in 2021. Journal: Biomed Res Int.

Not only in animal experiments but also in clinical studies, ICAM-1 has also been shown to be associated with ischemic stroke. A study in Finland showed that the expression of ICAM-1 was significantly upregulated after AIS, and it worked in concert with chemokines to cause granulocyte infiltration. This may be one of the potential mechanisms of ICAM-1 aggravating the neurological damage in stroke [41]. Unlike the above study, a clinical study in Croatia showed that serum ICAM-1 levels have nothing to do with the severity of stroke [42]. The explanation for this completely different conclusions may be as follows: first, the difference of race and second, the Croatian study is grouped according to different stroke subtypes, which may be the main reason for the different conclusions from the Finnish study. The results of Enlimomab Acute Stroke Trial Investigators showed that anti-ICAM-1 treatment not only failed to reduce the neurological damage of ischemic stroke but also significantly worsened the stroke outcome [43]. Interestingly, a recent study from China showed that serum ICAM-1 levels in AIS patients were elevated, and it was related to the increased risk of hemorrhage conversion after AIS [44].

Our research has some limitations. Firstly, our AIS patients come from a single center, and the sample size is small. Secondly, we have not dynamically monitored the changes in serum ICAM-1 nor have we conducted long-term follow-up of AIS patients. Thirdly, our AIS patients do not include patients treated with recombinant plasminogen activator (rtPA) and healthy volunteers. Therefore, we cannot evaluate the correlation between ICAM-1 and prognosis in patients with AIS after intravenous thrombolysis. Fourthly, we did not detect the levels of serum traditional inflammation markers nor did we explore their correlation with ICAM-1. Finally, we did not perform subgroup analysis of AIS patients with different causes. However, our research still has obvious advantages. Our study reported for the first time the correlation between serum ICAM-1 levels and the short-term prognosis of AIS stroke.

The article "Serum ICAM-1 as a Predictor of Prognosis in Patients with Acute Ischemic Stroke" was published in 2021. Journal: Biomed Res Int.

## 5. Conclusions

The level of serum ICAM-1 in AIS patients with poor prognosis was significantly higher than that in the good prognosis group. The baseline serum ICAM-1 level predicts the prognosis of AIS with high sensitivity and specificity. And after adjusting for multivariate, the serum ICAM-1 level is still an independent predictor of AIS functional outcome. The study of stroke targeting ICAM-1 is currently controversial, and more studies are still needed in the future to clarify this complex pathological mechanism.

## Figures and Tables

**Figure 1:** ROC analysis for the serum ICAM-1 level in the AIS patients.

**Table 1:** Characteristics of AIS patients with poor outcome and good outcome.

	Good outcome (*n* = 181)	Poor outcome (*n* = 105)	*p* value
Age, years	61.4 ± 8.9	61.7 ± 9.6	0.790
Male, *n* (%)	110 (60.8)	62 (59.0)	0.774
NHISS on admission	5 (2-7)	10 (8-14)	<0.001
Hypertension, *n* (%)	89 (49.2)	53 (50.5)	0.832
Diabetes mellitus, *n* (%)	54 (29.8)	32 (30.5)	0.909
Coronary heart disease, *n* (%)	19 (10.5)	12 (11.4)	0.807
Atrial fibrillation, *n* (%)	10 (5.5)	6 (5.7)	0.946
Systolic blood pressure, mmHg	148.3 ± 10.2	148.5 ± 10.7	0.875
Diastolic blood pressure, mmHg	92.6 ± 7.9	92.8 ± 8.3	0.840
Fasting blood-glucose, mmol/l	6.2 ± 0.8	6.3 ± 0.9	0.332
Total cholesterol, mmol/l	4.7 ± 1.2	4.8 ± 1.1	0.484
ICAM-1, pg/ml	117.5 ± 12.1	144.2 ± 14.8	<0.001

AIS: acute ischemic stroke; NIHSS: National Institute of Health Stroke Scale; ICAM-1: intercellular adhesion molecule-1.

**Table 2:** Risks variables for poor outcome at 3 months in AIS patients.

	OR	95% CI	*p* value
Age, years	1.35	0.843-1.418	0.231
Male, *n* (%)	1.16	0.902-1.194	0.365
NHISS on admission	0.65	0.436-0.803	0.058
Hypertension, *n* (%)	1.33	0.887-1.379	0.272
Diabetes mellitus, *n* (%)	1.31	0.835-1.352	0.107
Coronary heart disease, *n* (%)	1.18	0.891-1.205	0.329
Atrial fibrillation, *n* (%)	1.24	0.858-1.287	0.353
Systolic blood pressure, mmHg	1.35	0.774-1.386	0.432
Diastolic blood pressure, mmHg	1.31	0.970-1.361	0.504
Fasting blood-glucose, mmol/l	1.27	0.859-1.304	0.766
Total cholesterol, mmol/l	1.20	0.831-1.275	0.520
ICAM-1, pg/ml	0.52	0.318-0.839	0.007

AIS: acute ischemic stroke; NIHSS: National Institute of Health Stroke Scale; ICAM-1: intercellular adhesion molecule-1.

## Data Availability

The data used to support the findings of this study are available from the corresponding author upon request.
